# Effects of Fluid Shear Stress on Human Intervertebral Disc Nucleus Pulposus Cells Based on Label-Free Quantitative Proteomics

**DOI:** 10.1155/2022/3860898

**Published:** 2022-09-14

**Authors:** Liang-yu Xie, Sheng-nan Cao, Zi-teng Li, Dan-dan Wang, Bin Shi

**Affiliations:** Bone Biomechanics Engineering Laboratory of Shandong Province, Shandong Medicinal Biotechnology Center (School of Biomedical Sciences), Neck-Shoulder and Lumbocrural Pain Hospital of Shandong First Medical University, Shandong First Medical University, Jinan, Shandong Province, China 250062

## Abstract

**Objective:**

To explore the possible mechanism of fluid shear stress on human nucleus pulposus cells based on label-free proteomics technology.

**Methods:**

The human nucleus pulposus cell line was purchased and subcultured in vitro. The Flexcell STR-4000 multiflow field cell fluid shear stress loading culture system was used to apply continuous laminar fluid shear stress (12 dyne/cm^2^, 45 mins) to the monolayer adherent cells. Those without mechanical loading were used as the control group, and those subjected to fluid shear loading were used as the experimental group. Differential protein expression was identified using mass spectrometry identification technology, and bioinformatics analysis was performed using Gene Ontology GO (Gene Ontology) and Kyoto Encyclopedia of Genes and Genomes KEGG (Kyoto Encyclopedia of Genes and Genomes).

**Results:**

The proteomics results of the experimental group and the control group showed that the total number of mass spectra was 638653, the number of matched mass spectra was 170110, the total number of identified peptides was 32050, the specific peptide was 30564, and the total number of identified proteins was 4745. Comparing the two groups, 47 proteins were significantly differentially expressed, namely, 25 upregulated proteins and 22 downregulated proteins. Bioinformatics analysis showed that significantly different proteins were mainly manifested in cellular process, biological regulation, metabolic process, binding, catalytic activity, cellular components (cell part), organelle part (organelle part), and other molecular biological functions.

**Conclusion:**

Using proteomics technology to screen human nucleus pulposus cells after fluid shear stress loading, the differential protein expression provides a basis for further exploration of the mechanism of mechanical factors on nucleus pulposus.

## 1. Introduction

Intervertebral disc degeneration (IVDD) is a common clinical symptom and one of the important causes of low back pain [1]. According to epidemiology, the global prevalence of low back pain is 7.3%, and there are about 540 million people every day who are suffering from lower back pain [2]. It seriously affects the normal work and life of patients and brings a heavy economic burden to individuals and society. Aging, trauma, genetics, and biomechanical factors can influence the progression of IVDD [3]. The intervertebral disc itself is affected by various mechanical stimuli, such as pressure, tension, and shear stress [4]. Different stress magnitudes, frequencies, and stress time have various effects on the intervertebral disc [5]. Mechanical stress itself has twin effects, and ordinary stress stimulation will have an effect on the normal physiological structure of the intervertebral disc and the internal microenvironment of the intervertebral disc, thereby accelerating the process of intervertebral disc degeneration, while appropriate mechanical stimulation can regulate the synthesis of extracellular matrix that is conducive to retaining the intervertebral disc itself. McMillan, Garbutt, and Adams [6] studied the loading of the human lumbar intervertebral disc and found that continuous loading reduces the fluid content of the intervertebral disc, and proper exercise can promote the water circulation in the nucleus pulposus [7].

The NP consists of a massive quantity of proteoglycan and type II collagen. It can shape a completely unique porous machine, and the flow of fluid inside the nucleus pulposus will have an effect on the change of vitamins and affect the anabolism and catabolism of materials. Within the early stage, our study group established a fluid-structure interaction numerical strain model through finite element analysis and used the pressure acquisition system to collect the load parameters of the subjects on the L4/L5 lumbar vertebrae during the 3-dimensional balance spine manipulation manner and amassed the lumbar backbone geometry data of regular humans.

Mimics 21.0 and 3-Matic were built 3D computational modeling and found that when the intervertebral disc tissue is subjected to tensile stress, the inflow and outflow of water in the NP will be triggered [8]. It has been reported that the pressure on the intervertebral disc can be converted into fluid shear stress inside the nucleus pulposus [9]. Excessive fluid shear stress can promote the increase of inflammatory factor secretion and affect the expression of anabolic- and catabolic-related proteins. As a not unusual mechanical form within the human body, the effect of fluid shear stress on human intervertebral disc nucleus pulposus cells involves the conversion of mechanical factors to biochemical factors, but the mechanical target and molecular mechanism of fluid shear stress acting on the intervertebral disc are still not clear, and further research is needed.

In this study, by creating a fluid stress environment for human NP cells and using proteomics technology to detect the expression of differential proteins after fluid shear stress loading, it is beneficial to explain the influence of mechanical effect on the intervertebral disc nucleus pulposus cells.

## 2. Materials and Methods

### 2.1. Experimental Materials

Human normal nucleus pulposus cells (Wuhan Proser Biotech Biotechnology Corporation, China, batch number: CP-H097), fetal bovine serum (Gibco, USA, batch number: A3161001C), collagenase type II (Beijing Soleibo Technology Biotechnology corporation, China, batch number: C8150), 0.25% trypsin solution (Gibco, USA, batch number: 25200056), DMEM high-glucose liquid medium (HyClone, USA, SH30024.01), BCA protein quantification kit (Biyuntian Biotechnology Corporation, batch number: P0012), SDS-PAGE protein loading buffer (Biyuntian Biotechnology Corporation batch number: P0015F), iodoacetamide (IAA, batch number: I1149-5G), formic acid (Thermo Fisher Scientific, batch number: A117), trifluoroacetic acid (TFA, Sigma, batch number: T6508), and acetonitrile (Merck, batch number: 1000304008) are the experimental materials.

### 2.2. Experimental Apparatus

Fluid shear stress device STR-4000 (Flexcell, USA), NanoElute chromatograph-y system (Bruker, Bremen, Germany), Agilent 1260 Infinity II HPLC system, low-temperature high-speed centrifuge (Eppendorf 5430R), electrophoresis (BIO-RAD), Votex shaker (GENIE Votex-2), NanoDrop (Thermo Fisher Scientific ND2000), timsTOF Pro mass spectrometer (Bruker, Bremen, Germany), Multiskcan FC microplate reader (Thermo Fisher Scientific) (Taicang Huamei LNG-T98), MP Fastprep-24 homogenizer (MP Fastprep-24 5G), constant temperature incubator (Shanghai Jinghong, GNP-9080), and electronic balance (OHAUS AX324Z) are the experimental apparatus used for this study.

### 2.3. Cell Climbing

The nucleus pulposus cells were removed from liquid nitrogen and thawed. When the confluent density reached 85%–90%, the cells were washed with PBS. The NP cells were then dispersed using 0.25% trypsin (Gibco, USA) and resuspended in the appropriate culture plates. The cells were centrifuged at 1000 rpm for 5 min. Cell pellets were collected. 2–5 × 10^5^ cells were seeded on 75 × 25 × 1 mm glass slides and then allowed to stand at room temperature for 3 hours. The NP cells were transferred to the culture, and the experiment was started when the cells grew to 85% confluence.

### 2.4. Creation of the In Vitro Fluid Environment

Multiflow field cells were examined in cultured cells loaded with fluid shear stress. The quick interface should be connected exactly. Fluid passages are not bent and sterilized with alcohol. With PBS perfusion, the fluidic tubing was kept moist. 2% complete medium was used as the perfusate for mechanical loading. Slides overgrown with cells were transferred into fluid chambers. The dampers were tilted to reduce air bubbles.

### 2.5. Protein Extraction and Enzymatic Hydrolysis

Switching the glass slide to a square petri dish with a diameter of 100 mm, 0.25% trypsin was dropped to absolutely cover the floor of the glass slide. Allowing it to stand for 1 minute, the same amount of complete medium was set to terminate the digestion. Centrifuging at 1500 rpm for 5 minutes, the supernatant was collected. Uploading the right amount of SDT lysis buffer, we took a boiling water tub for 15 minutes and then centrifuged it at 14000 g for 15 minutes.

The BCA was used to quantify the protein in the control and experimental groups. Two groups of samples were taken 20 *μ*g each; added to 6× loading buffer, respectively; bathed in boiling water for 5 min; and subjected to 12% SDS-PAGE electrophoresis (constant pressure 250 V, 40 min), and Coomassie brilliant blue staining was used for quality detection. 80 *μ*g of protein solution was taken from each of the experimental group and the control group for FASP enzymatic hydrolysis, and DTT was added to the final concentration of 100 mm, and the solution was boiled for 5 min.

Adding 200 *μ*l of UA buffer, mixed well, we transferred it to a 30 kD ultrafiltration centrifuge tube. Adding 100 *μ*l of IAA buffer, the cells were set at room temperature in the dark for 30 min and centrifuged it at 12500 g for 15 min. Adding 100 *μ*l UA buffer and centrifuging it at 12500 g for 15 min, we then added 100 *μ*l of 40 mm NH4HCO3 solution and centrifuge at 12500 g for 15 min. We changed to a new EP tube, added 40 *μ*l trypsin buffer, shook it at 600 rpm for 1 min, and placed it at 37°C for 16–18 h. Adding 20 *μ*l of 40 mm NH4HCO3 solution, we collected the filtrate. The protein was desalted, and the lyophilized protein was reconstituted with 40 *μ*l of 0.1% formic acid solution, and the amount of protein at a wavelength of 280 nm was determined using a microplate reader.

### 2.6. Detection of Proteomics

The nucleus pulposus cells of the experimental group and the control group were detected by 4D label-free proteomics technology (Shanghai Jikai Gene Technology Biotechnology corporation), through protein extraction, protein quantification, SDS-PAGE, and protein enzymatic hydrolysis. The samples that passed the quality control were subjected to formal experiments using a high-resolution mass spectrometer to collect the original mass spectrometry data. According to the source of the sample, a specific protein database was built. Database matching was performed using Maxquant to obtain qualitative results of the protein, and FDR principle was used for data screening. Fisher's exact test was used to determine whether the differentially expressed proteins had a significant enrichment trend in certain functional types.

## 3. Results

### 3.1. Protein Mass Spectrometry Identification

The experimental group and the control group were subjected to analysis after enzymatic hydrolysis. The peptides detected by mass spectrometry were mainly distributed in 7–20 amino acids, which conformed to the general rule based on trypsin enzymatic hydrolysis and HCD fragmentation. The results showed that the total number of peptides measured in the experimental group. The control group was 638653. The number of matching peptides was 170110, and the number of specific peptides in the two groups was 30564. The total number of identified proteins was 4745. The relative molecular mass of proteins is concentrated in 5–100 kDa, accounting for 80% of the total number of proteins. There are 2141 proteins whose coverage is less than 20%, accounting for about 70% of the total number of proteins; 1029 proteins whose coverage is between 20% and 40%, accounting for 28% of the total number of proteins; and 443 proteins whose coverage is more than 40% occupied 12% of the total protein.

### 3.2. Statistics of Differential Proteins

Using proteomics technology to detect the experimental and control groups, a total of 47 DEPs were found. Compared with the control group, 25 DEPs in the experimental group were upregulated and 22 were downregulated (Tables 1 and 2). The difference in expression abundance of DEPs in the loading group and the control group can be seen by cluster analysis of differential expression (Figure 1).

### 3.3. GO Functional Annotation Analysis of Differentially Expressed Proteins

Map DEP to each GO entry in the GO database and count the number of upregulated and downregulated proteins under each GO secondary entry. 41 of the upregulated and downregulated proteins were mainly concentrated in cellular processes, 36 in biological regulation, and 35 in metabolic processes. 46 of the upregulated and downregulated proteins were concentrated in binding, and 22 differential proteins were concentrated in catalytic activity. 47 of the upregulated and downregulated proteins were concentrated in cellular composition, and 37 were concentrated in organelle composition (Figure 2).

### 3.4. GO Enrichment Analysis of Differentially Expressed Proteins

Blast2Go (https://www.blast2go.com/) software was used to perform GO functional enrichment analysis on the obtained differentially expressed proteins. The differentially expressed proteins can be obtained in BP, MF, and CC. Among them, there are top 10 in BP, such as keratinization, epidermal development, adhesion between endothelial cells, peptide cross-linking, regulation of tumor necrosis factor, lung development, negative regulation of vascular endothelial cells, cytoplasmic calcium ion transport, chondrocyte differentiation, and cell envelope organization. There are top 10 in MF, such as fibronectin binding, heparin binding, insulin-like growth factor binding, signaling receptor activator activity, protein glutamine gamma glutamyl transferase, extracellular matrix binding, calcium ion binding, structural composition of extracellular matrix, fibrinogen binding, and protein lysine 6 oxidase activity. There are top 10 in CC, such as basement membrane, keratinized envelope, fibrinogen complex, core binding factor complex, delta-DNA polymerase complex, BRCA1-BARD1 complex, extracellular matrix, integrin complex substances, sarcoplasmic reticulum, and insulin-like growth-binding protein (Figure 3).

### 3.5. Differential Protein KEGG Pathway Enrichment Analysis

Differential proteins are sorted in the pathway. The differential protein KEGG pathway annotation mainly includes metabolic pathways, biosynthesis of secondary metabolites, P13K-AKT signaling pathway, human papillomavirus infection, sphingolipids signaling pathway, AMPK signaling pathway, AGE-RAGE signaling pathway, and MAPK signaling pathway (Figure 4).

## 4. Discussion

The NP cells of the intervertebral disc faced complex mechanical load stimulation for a long time, and the mechanical stimulation can affect the structure and function of the intervertebral disc and the microenvironment inside the intervertebral disc. Our team found that the use of MechanoCulture FX2 like to load periodic stretch microstrain and found the stress of 100000 *μ*, 10% like tensile strain, frequency of 0.1 Hz, and 8640 cycles. It can significantly promote degenerated NP cell proliferation, inhibit the cell apoptosis, and promote the progression of the cell cycle [10]. Wang, Jie, and Jiwei [11] used low-, medium-, and high-frequency (3%, 9%, 19%) mechanical strains. They found that facing low-frequency mechanical strains and collagen type II and proteoglycan had no obvious effect. There were significant differences in increasing the expressions of TNF-*α*, IL-1*β*, and IL-6. The study showed that the effects of medium- and high-frequency mechanical strains were obvious. The results evidenced that low-frequency and high-frequency mechanical strains could promote intervertebral disc degeneration and the secretion of inflammatory factors through NF-*κ*B p65. Chao, Ma, and Ma [12] found that low-intensity stretch stimulation had a positive significance in anti-inflammatory response. Wang, Yang, and Hsieh [13] used alginate gel to simulate the internal environment of the nucleus pulposus, while showing that there is continuous fluid flow inside the NP under cyclic stress conditions.

Cao et al. applied moderate fluid shear stress to the immortalized nucleus pulposus cells. The study found that the strength was 12 dyne/cm^2^ and the loading time was less than 3 hours. The sGAG content and the aggrecan protein level were significantly increased, and the MMP13 protein level was significantly decreased. Fluid shear stress could slightly increase COL2a1 expressions and decrease ADAMTS5 expressions. Yichun et al. [14] found that when the strength of fluid shear stress is ≤12 dyne and the loading time is ≤45 minutes, the expression of BAD, Bax, and Caspase3 genes can be reduced in NP cells. As a special mechanical form, fluid shear stress can affect the proliferation, cycle, and apoptosis of various cells such as osteoblasts, osteoclasts, and chondrocyte-related phenotypes [15–17].

By creating a fluid shear stress environment for NP cells, this project used proteomics technology to screen the differential proteins between the experimental group and the control group. The results found that fluid shear stress can affect CCN1, DSG1, S100A7, THBS1, PTMA, KPRP, CNBP, and other proteins. Among them, CCN1 belongs to a member of the CCN family of stromal cell proteins, which is widely distributed in the extracellular matrix and is associated with various phenotypes such as cell proliferation, differentiation, senescence, and apoptosis. CCN1 has a significant role in promoting angiogenesis, and CCN1 exists in the embryonic mesenchymal layer during chondrogenesis and can promote chondrogenesis [18]. As a secreted matrix protein, CCN1 which can be affected by a variety of stimuli such as regulatory growth factors, cytokines, plasminogen, glycation end products, blood flow shear stress, and hypoxia. S100 protein, which exists in the cytoplasm or nucleus of various cells, can regulate cellular processes such as cell cycle and cell differentiation. Studies have found that compressive and shear mechanical stress can significantly upregulate the mRNA and protein levels of S100A7 and promoted resorption by inducing osteoclast differentiation and activity [19]. Relevant literature also showed that S100A7 can be affected by reactive oxygen species and played a role in the process of oxidative stress. Reactive oxygen species can induce the secretion of S100A7 [20]. THBS1 (thrombospondin-1) is an adhesion glycoprotein that mediates cell-to-cell and cell-to-matrix interactions, and it interacts with fibrinogen, fibronectin, laminin, type V collagen, and alpha-V/*β*-1 integrin binding. THBS1 had been extensively studied in renal, myocardial, and hepatic fibrotic diseases and had been found to play an important role in various ophthalmic diseases, namely, dry eye, ocular allergy, angiogenesis, lymphangiogenesis, wound healing, corneal transplantation, and infection. It has been reported that THBS1 can inhibit the formation of new blood vessels through various pathways [21]. The change of biomechanical load directly affected the metabolism of IVD cells, which has been widely regarded as an important factor leading to IVDD. Numerous studies had also proved that IVDD is involved in the formation of new blood vessels [22].

Our group previously found that applying tensile stress to the degenerated nucleus pulposus, mechanical loading form could mediate the proliferation of nucleus pulposus cells through P13K-AKT. The P13K-AKT signaling pathway is an intracellular signal transduction pathway that promoted metabolism, proliferation, cell survival, growth, and angiogenesis. The signal transduction mechanisms of the TGF-*β* family are controlled at the extracellular level, which include ligand secretion, deposition into the extracellular matrix, and activation [23]. Homologous recombination (HR) is a complex biological process that plays an important role in meiosis and repair of DNA double-strand breaks. The TGF-*β* signaling pathway is vital for the occurrence and growth of IVD and can play a protective role in the repair of IVD tissue by stimulating matrix synthesis, inhibiting matrix catabolism, inflammatory response, and cell loss.

Overactivation of TGF-*β* signaling was detrimental. When it was inhibited, TGF-*β* signaling can delay IVDD. Mechanical loading promoted the activation and release of TGF-*β* with integrins. TGF-*β* signaling promoted ECM synthesis in addition to inhibiting ECM in IVDD, promoting cell proliferation and inhibiting cell death [24]. AMPK acted as an important intracellular energy sensor, and its activity was regulated by energy imbalance, such as hypoxia, blood supply disturbance, and glucose deficiency. AMPK-induced autophagy promotes ECM synthesis and inhibits ECM degradation by regulating the expression of anabolic genes COL2A1, ACAN, and catabolic genes MMP-3, MMP-13, ADAMT-4, and ADAMT-5, thereby avoiding TBHP-induced autophagy and ECM destruction. AMPK further protects human NP cells from age-induced mitochondrial apoptosis by regulating SIRT3 [25].

In this study, proteomics was used to study the differential expression of proteins in the experimental group and the control group, and bioinformatics GO and KEGG analyses were used to reveal the functions of the differential proteins. In view of the characteristics of the protein itself, it can be used as a biomarker to explore biopathological processes [26]. The screening of differential proteins is the first step in the screening of protein markers. Subsequent verification of the screened differential proteins, as well as the enriched key proteins and star molecules of signaling pathways, can further clarify the effect of fluid shear stress on NP cells. In the near future, we will continue to develop this part. Proteomics technology was used to clarify the differential expression of proteins under mechanical action and to further clarify the effect and mechanism of fluid shear stress on nucleus pulposus cells. It has positive significance for clarifying the mechanical target of biomechanical stimulation on NP cells.

## 5. Conclusion

This is the first time we have used proteomic techniques to find the effects of fluid shear stress on NP cells. Based on the discovered differential proteins, we will further explore the mechanistic target.

## Figures and Tables

**Figure 1:** CTR1, CTR2, and CTR3 were the expression of differential proteins in the control group; Fss1, fss2, and fss3 are the differential protein expression of experiment group. Each column represents one sample, and each row represents the expression abundance of the same differential protein in different samples.

**Figure 2:** Column chart of differential protein GO notes.

**Figure 3:** Enrichment statistical bubble chart of the GO term (top 10).

**Figure 4:** The bubble diagram shows the KEGG pathway enrichment (top 20).

**Table 1:** Upregulated protein expression in both groups (top 10).

Number	Protein IDs	Gene name	FSS/CTR	*P* value	Regulation
1	O00622	CCN1	12.63	0.006	Up
2	Q02413	DSG1	7.73	0.014	Up
3	P31151; Q86SG5	S100A7; S100A7A	5.97	0.004	Up
4	P07996	THBS1	4.53	0.027	Up
5	P06454	PTMA	4.35	0.019	Up
6	Q5T749	KPRP	4.18	0.035	Up
7	P62633	CNBP	3.87	0.040	Up
8	Q9Y5Q0	FADS3	3.39	0.009	Up
9	Q14978	NOLC1	3.39	0.0001	Up
10	Q9NS91	RAD18	3.17	0.001	Up

**Table 2:** Downregulated protein expression in both groups (top 10).

Number	Protein IDs	Gene name	FSS/CTR	*P* value	Regulation
1	O60907	TBL1X	0.49	0.015	Down
2	O60507	TPST1	0.49	0.020	Down
3	P09972	ALDOC	0.48	0.022	Down
4	Q8NC96	NECAP1	0.48	0.002	Down
5	O00213	APBB1	0.48	0.023	Down
6	P06737	PYGL	0.47	0.022	Down
7	P98082	DAB2	0.47	0.003	Down
8	P49247	RPIA	0.47	0.007	Down
9	Q9NWM8	FKBP14	0.46	0.019	Down
10	Q7Z7L7	ZER1	0.46	0.006	Down

## Data Availability

The data used to support the findings of this study are available from the corresponding authors upon request.
